# The Importance of Cardiac Troponin Metabolism in the Laboratory Diagnosis of Myocardial Infarction (Comprehensive Review)

**DOI:** 10.1155/2022/6454467

**Published:** 2022-03-30

**Authors:** Aleksey M. Chaulin

**Affiliations:** Department of Cardiology and Cardiovascular Surgery, Department of Histology and Embryology, Samara State Medical University, Samara 443099, Russia

## Abstract

The study of the metabolism of endogenous molecules is not only of great fundamental significance but also of high practical importance, since many molecules serve as drug targets and/or biomarkers for laboratory diagnostics of diseases. Thus, cardiac troponin molecules have long been used as the main biomarkers for confirmation of diagnosis of myocardial infarction, and with the introduction of high-sensitivity test methods, many of our ideas about metabolism of these cardiac markers have changed significantly. In clinical practice, there are opening new promising diagnostic capabilities of cardiac troponins, the understanding and justification of which are closely connected with the fundamental principles of the metabolism of these molecules. Our current knowledge about the metabolism of cardiac troponins is insufficient and extremely disconnected from various literary sources. Thus, many researchers do not sufficiently understand the potential importance of cardiac troponin metabolism in the laboratory diagnosis of myocardial infarction. The purpose of this comprehensive review is to systematize information about the metabolism of cardiac troponins and during the discussion to focus on the potential impact of cTns metabolism on the laboratory diagnosis of myocardial infarction. The format of this comprehensive review includes a sequential consideration and analysis of the stages of the metabolic pathway, starting from possible release mechanisms and ending with elimination mechanisms. This will allow doctors and researchers to understand the significant importance of cTns metabolism and its impact on the laboratory diagnosis of myocardial infarction.

## 1. Introduction

Notwithstanding the solid achievements in the study of etiopathogenesis, diagnostics, and treatment of acute coronary syndrome, it still remains one of the leading reasons for disability and mortality of the population in all the developed countries of the world. All patients with acute coronary syndrome are under higher risk of the development of myocardial infarction and death [1–4]. According to the results of the reviews of myocardial infarction diagnostic criteria conducted in 2012 and 2018 by the European Society of Cardiology, the American College of Cardiology, the American Heart Association and the World Heart Federation, the diagnosis verification is based on the presence of myocardial ischemia symptoms (clinical, electrocardiographic, echocardiographic, and angiographic) and the positive dynamics of cardiac troponin levels in blood of patients [5–7].

Troponins (troponin I, troponin T, and troponin C) are proteins being a part of the troponin complex, which is bound to the protein tropomyosin. Tropomyosin, in its turn, together with actin, forms thin filaments of myocytes—the most important component of the contractile apparatus of striated muscle cells (of skeletal and cardiac muscles). All the three troponins participate in calcium-dependent regulation of the striated muscle contraction-relaxation. Each troponin type fulfils specific regulatory functions in contraction-relaxation of striated muscles. Troponin I is the inhibitory subunit of the tropomyosin complex that binds actin during relaxation and inhibits the ATPase activity of actomyosin thus preventing muscle contraction in the absence of calcium ions in the cell cytoplasm. Troponin T is the regulatory subunit, anchoring the troponin complex to thin filaments and, therefore, participating in the calcium-regulated contraction. Troponin C is the calcium-binding subunit. When the action potential is transferred to the muscle cell, calcium channels in the sarcoplasmic reticulum (“the repository of calcium ions”) open and the sarcoplasmic reticulum releases calcium ions into the sarcoplasm. Then, calcium ions bind to troponin C, which leads to the conformational (structural) changes of proteins of the troponin-tropomyosin complex, as a result of which the tropomyosin molecule shifts and releases binding sites for the myosin head on the actin filament. It enables the interaction of the myosin head with actin, which underlies the mechanism of contraction of striated muscles [8–11].

Molecules of troponins have a different amino acid structure depending on their localization in muscles, on the basis of which troponin isoforms are distinguished. Thus, troponin I has three isoforms: cardiac troponin I, troponin I of fast-twitch skeletal muscle fibers, and troponin I of slow-twitch skeletal muscle fibers. Troponin T also has three main isoforms: cardiac troponin T, troponin T of fast-twitch skeletal muscle fibers, and troponin T of slow-twitch skeletal muscle fibers. According to molecular genetic studies, the amino acid sequence of cardiac troponin I and cardiac troponin T differs from the amino acid sequences of the corresponding isoforms of skeletal troponins localized in skeletal muscle fibers by approximately 40-60% [12, 13]. This important structural peculiarity allows for the use of cardiac troponins T and I as specific biomarkers for laboratory diagnostics of myocardial injury in myocardial infarction and other noncardiac pathological conditions. Cardiac troponin C, as opposed to troponins I and T, has completely identical amino acid structure with the muscular (skeletal) troponin C, and increased blood levels of this protein will not let us reliably distinguish the cardiac muscle tissue injury from the damage of skeletal muscles, and, therefore, cardiac troponin С cannot be used as a cardiac marker for myocardial infarction diagnostics [14, 15].

Although the regulatory documents concerning the diagnostics and treatment of different forms of acute coronary syndrome and myocardial infarction contain clear recommendations on the time of troponin testing and decision-making levels, and the sensitivity and specificity of most immunoassays approximates 100%, there still remains a number of unsolved problems and issues relating to the application of these markers in clinical practice. Some of these problems are connected with the variety of troponin diagnostic agents, their unequal sensitivity and diagnostic accuracy, different susceptibility to cross-reactive substances (molecules), i.e., with different analytical characteristics of test systems [14, 16, 17]. Another range of issues results from the fact that the increase in cardiac troponin levels takes place in case of myocardial necrosis of any etiology and sometimes in the absence of irreversible myocardial injury (for instance, in case of reversible injury induced by physical exercises, renal failure, or the influence of false-positive factors) [18–24]. Besides, along with the necrosis of cardiomyocytes, there are other mechanisms of cardiac troponin release from myocardial cells and/or the increase in cardiac troponin concentration in blood serum. Thus, several clinical studies give evidence of very frequent increase in cardiac troponin concentration in various pathologies [24–28]. At the same time, the mechanism of troponin increase in these diseases is not associated with the ischemic necrosis of myocardial cells—the main mechanism of troponin levels increase in myocardial infarction. The study by Lindner et al. is quite representative in this respect. The researchers have conducted the detailed analysis of the reasons (the diseases) causing increase in cardiac troponin T levels in patients admitted to the emergency department. In total, the study included 1573 patients, and only 10% of which had the increased level of cardiac troponin T associated with myocardial infarction, while all the rest (about 90%) showed no signs of myocardial infarction, and their increased levels of troponin T were induced by other diseases causing the increase in troponin T serum levels by nonischemic mechanisms. The most common reasons of troponin T increase were the following ones: pulmonary embolism, renal failure, acute aortic dissection, heart failure, acute myocarditis, rhabdomyolysis, application of cardiotoxic chemotherapeutic agents, acute exacerbation of chronic obstructive pulmonary disease, sepsis and infiltrative cardiac pathologies (for example, amyloidosis). The interesting fact revealed by this study was that in 30% of cases the increased levels of troponin T were not connected with any previously described causes of cardiac troponin increase [25]. There is a high probability that these reasons might be connected with the false-positive mechanisms or they have been induced by the factors the researchers and medical practitioners have not paid attention to and have not described yet. Thus, the interpretation of the results showing the increased levels of cardiac troponins is an extremely complicated and sometimes even impossible task of modern clinical practice. Therefore, it is important to remember that the troponin test itself is not “the gold standard test” for myocardial infarction diagnostics, but it can become one only for those patients who show typical clinical symptoms of myocardial ischemia and have corresponding ischemic changes on the electrocardiogram, echocardiogram, etc. Generally, when interpreting possible reasons for the increase in cardiac troponins in blood serum, one should be guided by the following schematics (Figure 1).

Due to modern ultrasensitive tests, medical practitioners got the opportunity to early diagnose myocardial infarction (within the first two hours from admission of the patient) through the evaluation of dynamic changes of cardiac troponins. The changes (increase) of the concentration of cardiac troponin molecules within the first two hours are very small (may amount to as little as several ng/L) and cannot be detected by moderately sensitive test systems. It should be noted that due to a number of multicenter studies, there have been validated algorithms of early diagnostics (0 → 1 hour, and 0 → 2 hours) of non-ST-segment elevation myocardial infarction (NSTEMI) for ultrasensitive test systems of various manufacturers (Table 1) [29].

According to the data of modern (ultrasensitive) troponin test methods, the molecules of cardiac troponins are detected in blood and a number of other biological fluids in all healthy people [30–38], which poses new issues and challenges for the scientists in respect of search and explanation of possible mechanisms underlying the release of troponin molecules from intact myocardial cells. Hence, the molecules of cardiac troponins can be considered normal products of cardiac muscle tissue metabolism. However, the precise mechanisms of the release are not clear yet and are hypothetical. Moreover, the factors that may influence and facilitate or, on the contrary, reduce the release of troponins will be of great importance for researchers and medical practitioners. Currently, the most discussable biological factors influencing the degree of troponin release from healthy myocardium are the gender, age, and circadian characteristics [39–48]. Gender-related characteristics of cardiac troponins consist in the fact that the myocardium of healthy men releases more molecules of cardiac troponins than that of healthy women. These characteristics are validated by many clinical studies, and practically in all modern test systems, it is recommended to use the threshold values (99th percentile) in accordance with gender [41, 49, 50]. The age-related characteristics of cardiac troponins are that a greater amount of cardiac troponin molecules are released from the myocardium of elderly patients compared to the myocardium of young people [45, 51, 52]. The circadian features of cardiac troponins are that more cardiac troponin molecules are released from the myocardium of healthy people in the morning than from the myocardium of healthy people in the evening-night period [53, 54]. It should be noted that the age and circadian characteristics of cardiac troponins are not typical for all test systems, and according to some studies, they are contradictory [55–57]. Before using these characteristics in rapid diagnostic algorithms, it is necessary to conduct additional large studies to validate the age and circadian characteristics of cardiac troponins.

One of the significant problems of both moderately sensitive and modern highly sensitive immunoassays is the lack of their standardization [58–60]. This leads to the fact that different troponin immunoassays detect different values (concentrations) of cardiac troponin molecules in blood and other biological fluids of the same patient. So, in accordance with the data in Table 1, the threshold levels for excluding/confirming NSTEMI differ by several times when using immunoassays from different manufacturers [29]. Based on this, we can say that each method detects, in fact, different molecules of cardiac troponins and their fragments in a biological fluid. This creates certain difficulties and problems: (1) the need to validate the threshold concentrations of cardiac troponins for each test system, including newly developed ones, which is associated with additional high costs; (2) the need for a thorough study of interfering factors for each of the known detection methods that also involves additional costs; and (3) upon admission of a patient to the hospital, dynamic changes in cardiac troponins to confirm/exclude myocardial infarction during the first and subsequent hours can be traced and evaluated only when using the same test system, and immunoassays from different manufacturers cannot be used for this goal. At the same time, different institutions can use different test systems, which will not allow for proper assessment of the dynamic changes in case of urgently required transportation of a patient to another institution, which will be associated with a loss of time for additional examinations and additional economic costs.

It should be noted separately that the molecules of cardiac troponins can be affected by very numerous proteolytic enzymes present in blood, which thereby can indirectly affect the levels of troponins in blood of patients. For example, due to an increase in the activity of proteases that cause fragmentation of troponin molecules, the duration of circulation (half-life) of troponins in the bloodstream will decrease, which can potentially lead to false-negative results when using those test systems that have diagnostic antibodies directed against fragmented epitopes of troponin molecules [61, 62]. A decrease in the activity of such proteolytic enzymes, on the contrary, may hypothetically lead to false-positive results. However, the current specific knowledge about this metabolic stage, in particular, the exact information about all the influencing enzymes and mechanisms of troponin fragmentation, is extremely scarce and is not taken into account in clinical practice. This stage of troponin metabolism and its effect on diagnostics will be considered in more detail in this manuscript below in the paragraph on the circulation of cardiac troponins in blood plasma.

A very interesting direction in studying the diagnostic value of cardiac troponins is the assessment of the possibility of using other biological fluids as biomaterials for detection of troponin molecules. This direction is developing due to an increase in the sensitivity of immunoassays (the creation of highly sensitive and ultrasensitive test systems), which can detect very low concentrations (at levels of several ng/L) of troponins that circulate in many biological fluids, including noninvasively obtained fluids (urine and oral fluid) [34–47, 63–69]. Moderately sensitive methods, as a rule, cannot detect such low concentrations of cardiac troponin molecules present in these biological fluids [70, 71]. The mechanisms of penetration/transport of cardiac troponins into these biological fluids should also be considered as one of the stages of the metabolic pathway of cardiac troponins. And the study and understanding of precise mechanisms of penetration/transport of cardiac troponins will increase their diagnostic value and validate new methods for diagnosing cardiovascular diseases through the use of other biological fluids, in particular noninvasively obtained fluids, since their collection has a number of advantages (for example, painlessness and atraumatic nature, lower risk of introduction of blood-borne infections, and the possibility of obtaining biomaterial without the involvement of medical personnel) over the use of blood as a biomaterial. In addition, there are prospects for the creation of specialized diagnostic test strips (“dry chemistry” methods) for the detection of troponins in urine and/or oral fluid, which will make it possible to carry out express diagnostics and/or monitoring of cardiovascular diseases at home by patients themselves or by their relatives.

The main biological fluids in which the molecules of cardiac troponins are detected and their diagnostic value are summarized in Table 2.

### 1.1. Metabolic Pathway of Cardiac Troponins

Conventionally, there can be distinguished three main stages of the metabolic pathway of cardiac troponins (Figure 2): (1) release of cardiac troponins from myocardial cells, (2) circulation of cardiac troponins in blood plasma, and (3) removal of cardiac troponins from the bloodstream. Similar key stages of the metabolism of molecules are distinguished for other molecules in order to conveniently and consistently consider the main metabolic characteristics of molecules.

Each of these stages of metabolism can play a decisive role in the regulation of the concentrations of cardiac troponins in blood, i.e., their diagnostic value. In addition, there are a number of factors that can have a potential and hypothetical influence on these stages of the metabolic pathway of cardiac troponins. These factors can be physiological conditions, for example, gender, age, and circadian characteristics, which have a certain effect on the degree of release of troponin molecules from the myocardium of healthy people. Or, changes in the activity of proteolytic enzymes that target cardiac troponin molecules. The activity of proteolytic enzymes can also change under pathological conditions and/or in case of taking certain medications. Renal failure can be noted as an example of a significant factor affecting the removal of cardiac troponins from the bloodstream. It is important to emphasize that there may be an extremely large number of such factors, and some of them are probably still unknown.

Further in the course of this manuscript, I will sequentially consider each of the stages of the metabolic pathway of cardiac troponins and note the main known and assumed factors that may affect these mechanisms and the diagnostic value of cardiac troponins.

### 1.2. Release of Cardiac Troponins from Myocardial Cells: Mechanisms and Diagnostic Value

The introduction of highly sensitive test systems into practice made it possible with high accuracy (variability of the analysis within 10%) to detect very low concentrations of cardiac troponins, ranging from 0.001 to 0.01 ng/mL and below the values corresponding to the 99th percentile (upper limit of the norm). As a result, cardiac troponin molecules were found in almost 100% of healthy people, and instead of a clear borderline level typical of myocardial infarction, a smooth scale appeared, capable of reflecting subclinical myocardial pathology associated with structural (nonischemic) damage, stable coronary artery diseases and other pathological conditions that negatively affect myocardial cells [14, 38, 81–83]. Considering the fact that the molecules of cardiac troponins began to be detected in all healthy people, it became necessary to study and explain the mechanisms of the release of cardiac troponins from the intact myocardium. In this regard, the researchers are discussing the following possible mechanisms for the release of troponin molecules and an increase in their serum levels: a) the release of cardiac troponins as a result of the processes of regeneration and renewal of myocardial cells, b) the release of cardiac troponins as a result of apoptosis of myocardial cells, c) the release of cardiac troponins as a result of formation of membrane vesicles on the surface of myocardial cells, d) intracellular proteolytic degradation of cardiac troponin molecules into small fragments and the release of the latter through the intact membrane of myocardial cells, e) release of cardiac troponins as a result of the increase in the membrane permeability of myocardial cells, f) release of cardiac troponins as a result of small-scale (subclinical) necrosis of cardiomyocytes, g) the release of cardiac troponins from noncardiac cells. Some of the above mechanisms of release can not only explain the detectable concentrations of cardiac troponins in healthy individuals but also significantly activate/increase under certain physiological conditions and pathological processes [84–87]. For example, apoptosis of myocardial cells can increase with an increase in blood pressure [11, 88], stretching of the myocardial walls [89, 90], increased stimulation of beta-adrenergic receptors [91–93] and a number of other mechanisms [94, 95], which thereby may facilitate the release of cardiac troponins from cardiomyocytes. And in conditions of chronic renal failure, the expression of cardiac troponins in skeletal muscles is noted [96], which, according to some authors, can lead to an increase in serum concentrations of cardiac troponins in patients with chronic renal failure [96, 97].

Below, I will consider each of the above mechanisms of cardiac troponin release sequentially and in more detail.

### 1.3. Release of Cardiac Troponins as a Result of the Processes of Regeneration and Renewal of Myocardial Cells

Evidence of the fact that myocardial cells can regenerate/renew has been obtained by studying the metabolism of C^14^-labeled DNA molecules in myocardial cells. There was carried out a long-term observation of people with the inclusion of a radioactive isotope of carbon (C^14^) in the DNA of cardiomyocytes, which occurred as a result of nuclear weapons tests. The authors calculated the rate of renewal of cardiomyocytes by studying the rate of DNA synthesis, which was calculated by investigating the rate of accumulation of C^14^ in myocardial cells. There was found the renewal of cardiomyocytes, the intensity of which decreased annually—from 1% per year at the age of 25 years to 0.45% per year at the age of 75 years. In general, about 50% of cardiomyocytes underwent renewal throughout life [98, 99]. These results indicate the existence of a small regenerative potential in myocardial cells. Some researchers suggest that the process of renewal of myocardial cells may be associated with the release of cardiac troponins from cells [100]; however, the specific mechanism underlying this phenomenon remains unknown. As a possible hypothesis, it can be assumed that intracellular molecules of cardiac markers, including cardiac troponins, will be released from gradually aging and naturally dying cardiomyocytes as a result of the gradual destruction of the cell membrane. Since the rate of renewal of cardiomyocytes is low, the degree of increase in serum levels of cardiac troponins is also insignificant (no higher than the 99th percentile). Thus, this mechanism can hypothetically explain the presence of a small amount of cardiac troponin molecules in the bloodstream of all healthy individuals.

In accordance with the data of other researchers, the average rate of cardiomyocyte renewal in mammals is 0.5–2.0% per year and can vary depending on the influence of certain factors, such as physiological conditions (physical activity), trauma and concomitant diseases [101–103]. Thus, the rate of renewal of cardiomyocytes increases significantly after myocardial damage. An experimental study conducted by Docshin et al. has shown that ischemic myocardial injury causes the activation of endogenous stem cells and increases the rate of myocardial cell renewal [104]. Two other research groups led by Waring et al. [105] and Rovira et al. [106, 107] revealed an increase in the processes of proliferation and differentiation of stem cells in the myocardium of rats and zebrafish (Danio rerio).

However, the assessment of the degree of regeneration and the rate of renewal of myocardial cells can be significantly influenced by inflammatory processes, proliferation of nonmyocyte cells and the formation of a connective tissue scar in the myocardium, which often complicate and/or distort investigation results [108, 109]. Further research is needed to investigate the specific role of myocardial cell regeneration and renewal in the release of cardiac troponins from cells.

### 1.4. Release of Cardiac Troponins as a Result of Apoptosis of Myocardial Cells

To date, a large number of factors have been discovered that can trigger the processes of apoptosis of cardiomyocytes [110, 111]. Induction of apoptosis leads to an increase in the activity of caspases (proteolytic enzymes of the cysteine protease family), which can fragment (damage) DNA and protein molecules, leading to cell death. In contrast to necrosis, during apoptosis, the cell dies more slowly, the integrity of the cell membrane remains much longer, and the inflammatory reaction around the dead cell is not observed. To study the processes of apoptosis, many methods are used: various types of microscopy (light, electron, and fluorescence), flow cytometry, immunohistochemical analysis, the TUNEL method (terminal deoxynucleotidyl transferase (TdT) dUTP nick-end labeling), etc. The TUNEL method is the most reliable and early method for detecting apoptosis. This method allows visualization of cell nuclei in which the DNA molecule has been fragmented due to increased activity of endonucleases and caspases. This method is most often used in all modern studies aimed at the exploration of the etiopathogenetic mechanisms of apoptosis of various cells, including cardiomyocytes [112–114].

An experimental study led by Weil et al. has shown that short-term ischemia activates apoptosis of myocardial cells in experimental animals, and apoptosis of cardiomyocytes is accompanied by an increase in serum levels of cardiac troponins. Short-term myocardial ischemia was simulated by means of balloon occlusion of a branch of the left coronary artery and the fact of occlusion was confirmed by coronary angiography. The duration of ischemia was 10 minutes, after which reperfusion was carried out by deflation of the balloon. To confirm the apoptosis of myocardial cells, the TUNEL method was used, according to the results of which the number of cardiomyocytes in the state of apoptosis was significantly increased (6 times compared with the control group of animals). At the same time, no histological signs of myocardial necrosis were observed. This suggests that short-term (in this case, 10-minute) ischemia does not cause ischemic necrosis of cardiomyocytes, but enhances apoptotic processes in the myocardium. However, the levels of cardiac troponins began to rise rapidly: 30 minutes after reperfusion, the troponin I concentration approached the upper limit of the norm (38 ng/L) and after 1 hour exceeded it (51 ± 17 ng/L). Two and three hours after reperfusion, the serum levels of cardiac troponin I were 148 ± 88 ng/L and 180 ± 117 ng/L, respectively, which indicated the continuing release of troponin molecules from the myocardium. And, finally, 24 hours after reperfusion, the troponin I concentration reached its peak and amounted to 1021 ± 574 ng/L [115]. Thus, this experimental study elegantly demonstrates the role of apoptosis (induced by short-term ischemia) in the release of cardiac troponin molecules from myocardial cells. The limitation of this study is the relatively short interval of investigating the cardiac muscle tissue for the presence of histopathological changes; according to these results, it is impossible to determine the degree and reversibility of damage to cardiac myocytes during apoptosis induced by short-term ischemia. Besides, for detection of cardiac troponin I, there was used a moderately sensitive test system, which is inferior in diagnostic capabilities to modern highly sensitive immunoassays. In this regard, the dynamic changes in the levels of cardiac troponins detected by highly sensitive immunoassays during apoptosis could be significantly different, especially in the first minutes and hours after reperfusion.

The literature also describes other situations when apoptosis of cardiac myocytes is induced by other mechanisms that are not associated with reversible (short-term) ischemia of cardiac muscle tissue. The authors identify the following mechanisms of apoptosis that can promote the release of cardiac troponins from myocardial cells: stretching of the myocardial walls, increased preload on the heart, and increased activity of the sympathoadrenal system [89–91, 116]. Thus, Cheng et al. reported that apoptosis of myocardial cells increases with stretching of the myocardial walls [116]. This allows us to consider many physiological and pathological conditions that cause stretching of the myocardial walls as possible inducers of apoptosis and thus can, to some extent, explain the increased serum levels in patients after prolonged and intense physical exertion or having arterial hypertension, pulmonary embolism, chronic obstructive pulmonary disease and a number of other pathologies [116–119].

In another experimental study, Weil et al. concluded that an increase in preload on the heart triggers apoptosis and causes an increase in the concentration of troponin I in blood of experimental animals. To increase the preload on the heart, the experimental group of animals received intravenous drug—phenylephrine (300 *μ*g of the drug per minute) for one hour. After the simulation, echocardiography was used to confirm myocardial overload, and to verify apoptosis and determine cardiac troponin levels, there were used histological methods, including the TUNEL method and moderately sensitive immunoassay, respectively. As a result of histological examination of the myocardium of the experimental group of animals, there was noted a significant increase in the number of cardiomyocytes in the state of apoptosis, as compared to the control group. At the same time, no histological signs of myocardial necrosis were recorded. 24 hours after the simulation, the number of cardiomyocytes in the state of apoptosis decreased to the level of the control group, which indicates the reversibility of apoptotic changes. The troponin I concentration exceeded the upper limit of the norm 30 minutes after the simulation, and then the troponin I levels continued to rise sharply and reached a value of 856 ± 956 ng/L one hour after the simulation. Serum levels of cardiac troponin I remained elevated throughout the study period (24 hours) and peaked at 1462 ± 1691 ng/L [120]. Since signs of necrosis, unlike apoptosis, were not observed, it should be considered that apoptosis induced by myocardial overload plays an important role in the release of cardiac troponin molecules from cells [121].

The degree of release of cardiac troponin molecules from myocardial cells as a result of apoptosis induced by myocardial overload depends on the strength and duration of exposure. For example, relatively small myocardial overload is observed on mild to moderate exertion, in hypertension and nonmassive pulmonary embolism, so the increase in serum levels of cardiac troponins in these conditions is also relatively small. But, for example, on high-intensity exertion or in massive pulmonary embolism, myocardial overload becomes much more significant; therefore, these conditions are accompanied by relatively higher serum levels of cardiac troponins [122–124].

Another very interesting mechanism for the initiation of apoptosis is an increase in the activity of the sympathoadrenal system. A research group led by Singh et al. found that stimulation of beta-adrenergic receptors (*β*-AR) regulates intracellular apoptotic signaling pathways in cardiomyocytes. Moreover, stimulation of *β*1-AR enhances apoptosis of myocardial cells, while stimulation of *β*2-AR has the opposite effect [125, 126]. It was also noted that the density of *β*-AR subtypes changes significantly with age [127]. Thus, in elderly patients, a more pronounced decrease in the number of *β*2-AR is noted, which may contribute to a weakening of the anti-apoptotic effect and, accordingly, an increase in apoptosis of myocardial cells [127–129]. A higher degree of apoptosis in elderly patients can probably be associated with age-related characteristics of cardiac troponin levels: in older people, troponin levels are significantly higher than in young people. The age-related characteristics of cardiac troponins have been demonstrated in a number of clinical studies through blood examination with highly sensitive test systems [43–45, 51, 52].

Considering the above, apoptosis of cardiomyocytes should be considered as a significant mechanism for the release of cardiac troponin molecules from myocardial cells. This mechanism is not associated with necrosis of cardiomyocytes and contributes to a very significant increase in serum levels of cardiac troponins. Thus, apoptosis of myocardial cells can be of great diagnostic value in conditions such as prolonged and intense physical activity, arterial hypertension, pulmonary embolism, heart failure, and, probably, in old age. Further research is needed to clarify the exact role of apoptosis in the release of cardiac troponins in physiological and pathological conditions.

### 1.5. Release of Cardiac Troponins as a Result of the Formation of Membrane Vesicles on the Surface of Myocardial Cells

This mechanism of release of cardiac troponins from myocardial cells was first described in an experimental study relatively long ago. A research group led by P. Schwartz reported that on the plasma membrane of myocardial cells membrane vesicles (blebbing vesicles) are formed [130, 131]. And during ischemia, the number of blebbing vesicles increases in comparison with intact myocardial cells. A similar trend is also typical for hepatocytes [132]. Since these vesicles are formed from fragments of the cell membrane and the cytoplasm of cardiomyocytes, these vesicles may contain some cytoplasmic proteins of myocardial cells, in particular cardiac markers (creatine kinase MB isoform, myoglobin and the cytoplasmic fraction of cardiac troponins, and others). However, since the volume of the cytoplasmic fraction of cardiac troponins is small (approximately 3–4% for troponin I and 7–8% for troponin T of the total amount of troponins in the cardiomyocyte) [53, 133], the contribution of this mechanism to the degree of increase in serum levels of cardiac troponins will also be limited. Based on the peculiarities of the formation of blebbing vesicles (a significant increase in ischemia), it can be assumed that this mechanism is involved in the release of cardiac troponins in those pathological conditions that are accompanied by ischemia of myocardial cells at an early stage. For example, the initial (prenecrotic) stage of myocardial ischemia can provoke the formation of blebbing vesicles and the release of troponins into the bloodstream, which will lead to the formation of the first peak in serum concentrations of cardiac troponins. Subsequently, two main scenarios are possible: (1) with a decrease in ischemia of myocardial cells, the formation of blebbing vesicles stops and troponin concentrations quickly return to normal, and (2) with the continuation/intensification of ischemia (for example, during myocardial infarction), the formation of blebbing vesicles increases, and, in addition to this, there occurs the destruction of the plasma membrane of myocardial cells and proteolysis (fragmentation) of troponin proteins, which are part of the main (structural or contractile) troponin fraction, which will lead to the formation of the second peak in serum concentrations of cardiac troponins. From a pathogenetic point of view, any physiological or pathological condition that will lead to ischemia of myocardial cells (even reversible myocardial ischemia) can activate this mechanism of cardiac troponin release. For instance, some physiological conditions (physical activity) [134] or pathological conditions (sepsis) [135] can cause an increase in the oxygen demand of myocardial cells, which, accordingly, will be accompanied by ischemia of the cardiac muscle tissue.

## 2. Intracellular Proteolytic Degradation of Cardiac Troponin Molecules into Small Fragments and the Release of the Latter through the Intact Membrane of Myocardial Cells

The size and location of intracellular molecules are two key factors that affect the transport (release) of molecules across the cell membrane. Low molecular weight biomarkers are much more intensively released across the plasma membrane, which plays a role in the diagnostics of many diseases, including cardiovascular pathologies. So, for example, with the development of myocardial infarction, the concentration of low molecular weight cardiac markers (myoglobin) in blood serum rises much earlier than the concentration of high molecular weight cardiac markers (lactate dehydrogenase-1) [136–138]. This is due to the fact that myoglobin molecules are small and can be released at the initial stages of ischemia during the development of myocardial infarction (when the plasma membrane of myocardial cells is still relatively insignificantly damaged). A larger molecule (lactate dehydrogenase-1) can leave the cardiomyocyte only when its cell membrane is significantly damaged. Biomarkers that are freely localized in the cytoplasm of cells (for example, myoglobin and cytoplasmic (noncontractile) fraction of troponins) also have advantages when released from the cell, in contrast to those biomarkers that are localized in organelles (nucleus or mitochondria of cells) or are tightly bound to structural components of sarcoplasm (for example, the structural fraction of troponins involved in the regulation of the contractile fraction of the myocardium). So, during the development of myocardial infarction, the primarily released molecules are troponin molecules that are part of the cytoplasmic fraction of cardiac troponins, and only then there takes place the destruction of sarcomeres, in particular of the troponin-tropomyosin complex, and the release of structural cardiac troponins.

The most important factor that can affect the size of a molecule (biomarker) and, accordingly, the possibility of its release, is the degree of activity of enzymes that cause proteolysis (fragmentation) of this molecule [139, 140]. The activity of proteolytic enzymes can change both under physiological and pathological conditions. In an experimental study conducted by Feng et al., it was demonstrated that an increase in preload on cardiac muscle tissue activates the enzyme calpain, which fragments the cardiac troponin I molecule, which could potentially play a role in the release of this biomarker from myocardial cells and an increase in its level in blood serum [140]. Thus, physiological and pathological conditions causing an increase in the preload on the myocardial wall can promote the release of cardiac troponins from myocardial cells by this mechanism.

In addition to the enzyme calpain, the cleavage of cardiac troponin molecules can be catalyzed by some types of matrix metalloproteinases (MMP 2 and MMP 14) [140–143] and the enzyme thrombin [144–146]. The activity of these enzymes can also be influenced by pathological processes and some drugs, which thereby hypothetically can affect the serum levels of cardiac troponins. For example, an increase in thrombin activity in patients with dilated cardiomyopathy [147, 148] can contribute to the fragmentation of cardiac troponin T, which can have both pathogenetic significance (damage to troponin T, which is one of the main components of the contractile apparatus of cardiomyocytes), and diagnostic value: a decrease in the size of the troponin T molecule as a result of fragmentation and a possible increase in the release of these fragments into the bloodstream.

Changes in acidity (pH) can also modulate the activity of intracellular proteolytic enzymes [149, 150]. So, pathological conditions that disrupt myocardial metabolism, in particular myocardial ischemia, lead to a switch from aerobic myocardial metabolism to anaerobic metabolism and an increase in the formation of lactic acid, which will shift the pH towards acidosis. Under conditions of acidosis, then, proteolytic and proapoptotic enzymes will be activated [69, 140, 150, 151], which, through fragmentation, will promote the formation of many small fragments (molecules) of cardiac troponins, which will increase the likelihood of their release from myocardial cells into the bloodstream.

### 2.1. Release of Cardiac Troponins as a Result of Increased Membrane Permeability of Myocardial Cells

The membrane permeability of myocardial cells is an important factor that plays a role in the release of cardiac marker molecules from myocardial cells into the bloodstream. Based on the analysis of the results of existing experimental data, two main mechanisms can be distinguished that underlie the change (increase) in the membrane permeability of myocardial cells: (1) an increase in the membrane permeability of myocardial cells as a result of an increase in the load on the myocardium and stretching of its walls and (2) an increase in the membrane permeability of myocardial cells as a result of myocardial ischemia and activation of proteolytic enzymes that can damage the cell membrane.

The first mechanism for the release of cardiac troponins was studied by Hessel et al. [152]. In their experimental study, the authors stimulated special glycoprotein receptors of myocardial cells (integrins) that are sensitive to myocardial stretching. To model myocardial stretching and activation of integrins, the researchers used the RGD (Arg-Gly-Asp) tripeptide, which is a potent integrin agonist and is part of fibronectin and other regulatory proteins of the extracellular matrix [153]. The authors particularly note that myocardial stretching is not associated with ischemic and necrotic processes in the cardiac muscle tissue, which indicates that it was the specific mechanism of myocardial wall stretching and the activation of integrins that ensured the release of cardiac troponins from viable myocardial cells [152].

The second mechanism for increasing membrane permeability is associated with membrane damage during ischemia of myocardial cells. As already described above, myocardial ischemia initiates changes in the metabolism of cardiomyocytes and acidification (acidosis) of the intracellular space of myocardial cells, which, in turn, will lead to the activation of proteolytic and proapoptotic enzymes. These enzymes have many targets and in addition to the specific action (fragmentation of cardiac troponins), they can obviously catalyze the proteolysis of proteins that make up cell organelles and membranes [154–156]. Thus, this mechanism of troponin increase is closely interrelated with the above-described mechanism (troponin increase due to increased proteolytic degradation into small fragments). In general, increased membrane permeability and intracellular fragmentation of cardiac troponins can be considered as two interrelated and synergistic mechanisms underlying the release of cardiac troponin molecules from myocardial cells. The degree of activity of these mechanisms is probably related to the severity of pathological processes. For example, short-term and/or reversible ischemia of myocardial cells during exercise or in uncomplicated sepsis may be associated with a relatively small increase in the activity of intracellular proteolytic enzymes. In this regard, the degree of increase in serum levels of cardiac troponins will also be relatively small and dependent only on the cytoplasmic fraction of cardiac troponins (their fragmentation into small molecular fragments) and reversible membrane damage/increased membrane permeability. In pathological conditions that cause irreversible ischemia of myocardial cells (for example, myocardial infarction or severe/complicated sepsis), serum troponin levels increase much more significantly and the main contribution to total serum levels of cardiac troponins will be made by the structural fraction of cardiac troponins. Both the proteins of the troponin-tropomyosin complex and the proteins of the membranes of cardiomyocytes will be more actively fragmented (cleaved) and therefore the degree of release of cardiac troponins in these pathologies will be higher. The further prognosis of patients suffering from both cardiac and noncardiac pathologies is also associated with the degree of increase in serum levels of cardiac troponins, which indicates the depth and nature of damage to cardiac muscle tissue.

### 2.2. Release of Cardiac Troponins as a Result of Small-Scale (Subclinical) Necrosis of Cardiomyocytes

A possible mechanism underlying the release of cardiac troponins is small-scale necrotic processes, which can be caused by both ischemia and inflammatory-toxic processes, imbalances in the neurohumoral system.

So, according to some researchers, regular heavy physical exertion, myocarditis and stressful situations can cause subclinical damage to myocardial tissue (death of single cardiomyocytes), which can subsequently be associated with the formation of relatively small areas of fibrosis and an increased risk of sudden cardiac death [157]. So, for example, the adverse effect of serious and/or intense physical activity is confirmed by a number of studies and described clinical cases in which sudden cardiac death was recorded in athletes [158–160].

Some studies registered extremely high levels of cardiac markers, including cardiac troponins in the blood serum of athletes after serious and prolonged physical activity [161–163], which is also a reason for discussing possible small-scale necrotic processes. A contradictory argument is a clinical study using magnetic resonance imaging with gadolinium (contrast) that revealed no signs of necrosis and sclerosis in the cardiac muscle tissue of athletes [164]. However, the limitation of this method is its relatively lower sensitivity compared to laboratory biomarkers of myocardial necrosis and fibrosis.

Although during psycho-emotional stress the level of troponin increase is relatively small (rarely exceeds the levels of the 99th percentile in the isolated effect of stress), it cannot be considered a safe process [165, 166]. The constant influence of stress is considered as a risk of developing cardiovascular diseases and may be one of the triggers of myocardial infarction [167, 168]. A number of molecules released during stress (for example, cortisol and catecholamines) increase myocardial oxygen demand, thereby contributing to the development of relative ischemia of myocardial cells.

### 2.3. Release of Cardiac Troponins from Noncardiac Cells

One of the controversial but hypothetically possible mechanisms underlying the increase in serum levels of cardiac troponins is the release of these molecules from noncardiac cells. Several experimental and clinical studies indicate the expression of cardiac troponin molecules in skeletal muscle cells [96, 169, 170] and the walls of large vessels [171, 172], which allows us to consider these organs as possible sources of serum levels of cardiac troponins. Thus, American biochemists (Ricchiuti and Apple), using polymerase chain reaction (PCR), revealed the expression of messenger RNA of cardiac troponin T in the skeletal muscle tissue of adults suffering from end-stage chronic renal failure and hereditary skeletal myopathy (Duchenne muscular dystrophy). Cardiac troponin I messenger RNA was not detected in skeletal muscles of patients suffering from these pathologies and in skeletal muscles of healthy people. In addition, no signs of cardiac troponin T expression were detected in the skeletal muscles of healthy people [96], which indicates the possible expression of one type of cardiac troponin (T) only in the presence of the indicated pathologies. In another study, Messner et al. confirmed the possibility of extracardiac expression of cardiac troponin T in patients with skeletal myopathies. The researchers, using PCR, found messenger RNA of cardiac troponin T in patients with primary sarcoglycanopathy and Duchenne muscular dystrophy [170]. In some patients with skeletal myopathies, in addition to cardiac troponin T messenger RNA, the expression of cardiac troponin I messenger RNA was observed [170]. However, in these studies, the authors did not measure serum levels of cardiac troponins in patients with myopathies and renal failure. This is an important limitation of these studies because it does not answer the question: can the expression of cardiac troponins in skeletal muscles lead to an increase in serum levels of cardiac troponins in patients with chronic renal failure or hereditary skeletal myopathies? In addition, there should be mentioned several other studies, the results of which contradict the above data on noncardiac expression [173–176]. For example, Bodor et al. conducted a study and concluded that cardiac troponins are not expressed in skeletal muscle tissue in patients with Duchenne muscular dystrophy and polymyosites [173]. Other research groups led by Hammerer-Lercher and Schmid also did not find signs of expression of cardiac troponins in skeletal muscles [174].

A second potential noncardiac source of cardiac troponin release is the walls of large veins (venae cavae and pulmonary veins). Some studies report only the presence of expression of cardiac troponins in the walls of these veins, but do not describe the possible role of these troponins in diagnostics [171, 172]. Hypothetically, it can be believed that damage or stretching of the walls of these large veins can lead to the release of cardiac troponin molecules into the bloodstream.

Thus, due to the fact that data on extracardiac expression are either insufficient or contradictory, further research is needed to validate this mechanism.

The mechanisms of cardiac troponin release described above and their diagnostic value are summarized in Table 3.

### 2.4. Circulation of Cardiac Troponins in Blood Plasma: Influencing Factors and Diagnostic Value

The second major stage of the metabolic pathway of cardiac troponins is circulation in the bloodstream. At this stage, the molecules of cardiac troponins are influenced by a number of factors (activity of proteolytic enzymes, kinases, phosphatases, the state of renal function, and the reticuloendothelial system), which can affect serum levels of cardiac troponins and, therefore, their diagnostic value. The molecules of cardiac troponins released into the bloodstream are represented by a heterogeneous fraction (a significant variety of different forms of troponin molecules): free troponins; combined complexes consisting of several free forms of cardiac troponins (for example, cardiac troponin I+troponin C and cardiac troponin T+cardiac troponin I) and small fragments of cardiac troponins [61, 144, 145, 177–181]. All of the above forms of troponin molecules can undergo oxidation, glycosylation, phosphorylation and dephosphorylation processes, which leads to the formation of very diverse forms (varieties) of troponin proteins. Modifications of troponin proteins can affect such an important parameter as the half-life (half-decay) of cardiac troponins. This parameter has not only fundamental but also high practical importance, since with an intensification of the breakdown of troponin proteins, their concentration and the “diagnostic window” can decrease, and with a weakening of the breakdown of cardiac troponins, their serum levels and the duration of the diagnostic window can increase. The researchers estimate that the half-life of cardiac troponin T in the bloodstream is approximately 2 hours, however, for many other forms, the half-life is controversial and unknown [182–184]. The cardiac troponin I molecule is much less stable in the bloodstream, since it actively undergoes the processes of oxidation, phosphorylation and fragmentation [185–187]. The latter, in turn, as noted above for cardiac troponin T, depend on the activity of these enzymes, the presence of concomitant pathologies that can affect the activity of these enzymes, the intake of drugs that affect the catalytic activity of proteolytic enzymes and the functional state of the organs responsible for the elimination of molecules of cardiac troponins. For example, increasing the activity of the enzyme thrombin (which has been shown to cause specific fragmentation of cardiac troponin T) [145] can reduce the half-life of cardiac troponin T and its concentration in the bloodstream. It is logical that taking drugs that reduce thrombin activity (for example, direct thrombin inhibitors, direct and indirect anticoagulants) can increase the half-life of cardiac troponin T and the duration of the diagnostic window. As examples of the influence of other factors on the duration of the circulation of cardiac troponins in the bloodstream, there can be named the functional state of the kidneys and the reticuloendothelial system. Thus, protein molecules of cardiac markers, including cardiac troponins T and I, can be captured by the reticuloendothelial system (macrophages) and are destroyed there [67, 187, 188]. Based on this, the following point of view comes out: an increase in the activity of the reticuloendothelial system (for example, with hypersplenism and splenomegaly) may be accompanied by an increase in the cleavage of cardiac troponins and a decrease in the half-life; and a decrease in the activity of the reticuloendothelial system, on the contrary, will lead to a weakening of the cleavage of cardiac troponins and an increase in the half-life. Renal function is also significantly associated with cardiac troponin levels and increased blood protease activity. Thus, an increase in the activity of proteolytic enzymes can lead to the formation of a large number of small fragments of troponin molecules, which, like many low molecular weight proteins, can be filtered through the three-layer glomerular (filtration) barrier of nephrons. However, the filtration rate can change both under physiological and pathological conditions, which can have a significant effect on the rate of removal of troponin fragments. With pronounced drops in filtration rate (for example, with chronic renal failure or a decrease in blood pressure), the molecules of cardiac troponins will not be filtered (removed) from the bloodstream into the urine, but will accumulate in the blood, which will lead to an increase in the half-life of cardiac troponins and prolongation of the diagnostic window [189–191].

Clear evidence that cardiac troponin molecules can pass (filter) through the glomerular filter has been presented in several recent clinical studies due to the use of highly sensitive troponin immunoassays [34, 67, 69]. A similar transport mechanism is probably characteristic of the filtration of cardiac troponins into the oral fluid through the blood-salivary barrier, which is also supported by several pilot studies that have established a correlation between serum and salivary troponin levels [35–37, 68].

The search for specific mechanisms of proteolytic cleavage of cardiac troponins in the bloodstream is of great practical importance, since it will optimize laboratory diagnostics: in particular, there is a possibility of developing antibodies directed against individual fragments of cardiac troponins or introducing inhibitors of the main proteolytic enzymes that catalyze troponin proteolysis into diagnostic test systems to reduce interference and more thoroughly interpret the test results, taking into account comorbidities that affect the activity of enzymes breaking down cardiac troponins. Unfortunately, the number of fundamental studies devoted to the investigation of the processes of proteolytic cleavage of cardiac troponins in the bloodstream is extremely small. And to date, only one specific mechanism is known, described in the study by Katrukha et al. [61, 145]. According to the results of this study, the enzyme thrombin catalyzes the cleavage of the full-length molecule of cardiac troponin T (the molecular weight is 35 kDa) in the region of the peptide bond between amino acids 68 and 69 into two fragments, one of which is larger (the molecular weight is 29 kDa), and the second—smaller (the molecular weight is 6 kDa) [145]. As noted above, any significant effect on thrombin activity (for instance, the use of anticoagulants) can influence the fragmentation of troponin T and, accordingly, its diagnostic value.

In general, a number of research groups studying the processes of proteolytic cleavage in the bloodstream report the presence of a very large number of fragments (approximately several tens) of cardiac troponin molecules, which have different sizes (molecular weights from several kDa to 30 or more kDa), stability and half-life in the bloodstream (from several hours to a day) and conditions of formation (physiological conditions, the degree of severity and progression of ischemia, reperfusion time, etc.) [144, 145, 177–181]. Vylegzhanina et al. studied the composition of troponin complexes in patients with myocardial infarction [181]. The researchers have identified the following main forms of cardiac troponins in myocardial infarction: a ternary complex consisting of full-size cardiac troponins T and I and troponin C; a ternary complex consisting of truncated cardiac troponin I and integral troponins T and C; a binary complex consisting of truncated cardiac troponin I and troponin C, as well as a number of short fragments of cardiac troponin T and troponin I, formed mainly from the central part of the molecules. As AMI progressed, there was a decrease in the number of ternary complexes consisting of full-size cardiac troponins and an increase in the number of ternary and binary complexes consisting of truncated troponins, as well as an increase in the level of fragments of cardiac troponins [181]. Such changes in the heterogeneous fraction of cardiac troponins are most likely due to an increase in the activity of proteolytic enzymes, which increase with the progression of ischemia and myocardial infarction, and, accordingly, cause fragmentation (truncation) of troponin proteins.

Very interesting data are presented by the researchers Zahran et al., who studied the degree of proteolytic degradation of cardiac troponin I in patients with varying degrees of ischemia and damage to cardiac muscle tissue [180]. The researchers noted that the degree of proteolytic cleavage of cardiac troponin I increases with an increase in the severity of ischemia and myocardial injury: the highest degree of proteolytic cleavage of cardiac troponin I was characteristic of patients with ST-segment elevation myocardial infarction, while in patients with non-ST-segment elevation myocardial infarction the degree of troponin I degradation was significantly lower. The authors also found a decrease in the degree of proteolytic degradation of cardiac troponin I after reperfusion, which can probably be used to assess the quality of reperfusion. It is quite remarkable that the degree of proteolytic degradation of cardiac troponin I had a higher diagnostic value in myocardial infarction than the total serum concentration of cardiac troponin I [180].

Summing up the role of the stage of cardiac troponin circulation, we should once again emphasize its potentially high diagnostic value for practical medicine. At the moment, this stage is a relatively poorly studied area of the biology of cardiac troponins. The main directions of further work in this area, in my opinion, should be as follows:

1. Study of the fundamental specific mechanisms of proteolytic degradation of cardiac troponins in the bloodstream both under normal conditions and under the conditions of simulated concomitant pathologies. This requires a targeted and thorough study of the potential effect of individual serum proteolytic enzymes (for example, specific thrombin-mediated degradation of cardiac troponin T)
2. Search for specific fragments of cardiac troponins, which are released at the earliest possible time after the onset of myocardial ischemia and the creation of antibodies to them, which will increase the sensitivity and specificity of troponin immunoassays
3. Search for specific fragments of cardiac troponins, which have a small molecular weight and are able to pass through the glomerular and blood-salivary barriers. The creation of antibodies to these fragments will make it possible to develop specific highly sensitive test systems for the analysis of noninvasive biological fluids (urine and oral fluid) and for the introduction of new methods of noninvasive diagnostics and monitoring of cardiovascular pathologies, including myocardial infarction, into routine clinical practice
4. Study and identification of potentially possible specific mechanisms of proteolytic cleavage of cardiac troponins under the action of other (nonischemic) factors. This will allow the development of specific troponin immunoassays to identify those fragments that, for example, will increase exclusively with stretching of the myocardium or exclusively with an increase in the activity of the adrenergic nervous system and an increase in *β*-AR stimulation. Thus, it will be possible to carry out a more specific diagnosis of nonischemic myocardial damage in some physiological and pathological conditions not associated with ischemia of the cardiac muscle tissue

### 2.5. Removal of Cardiac Troponins from the Bloodstream: Mechanisms and Diagnostic Value

The final stage of the metabolic pathway of cardiac troponins in the bloodstream is as important as the other two stages (release and circulation). Both of these stages are closely related to the terminal stage of the metabolic pathway of cardiac troponins. So, for example, when small fragments are released from cardiomyocytes (as a result of intracellular proteolytic cleavage of cardiac troponins), they will obviously be almost immediately removed from the bloodstream by filtration through the glomerular and blood-salivary barriers. When larger fragments of cardiac troponins and/or binary and ternary complexes are released, filtration of these molecules is unlikely due to their large size (molecular weight).

The circulation of cardiac troponins is equally closely related to the removal of these molecules. So, for example, with a higher activity of serum proteolytic enzymes, the process of degradation of cardiac troponin molecules will be more active, which will lead to more rapid formation of small troponin molecules and their filtration (removal) from the bloodstream.

In general, today, the mechanism of filtering cardiac troponins through the glomerular barrier is one of the main and definitively proven ways to remove cardiac troponins from the bloodstream. The inferential (indirect) evidence is that when the filtration rate decreases (for example, in chronic renal failure), cardiac troponin molecules accumulate in the bloodstream and their serum levels begin to rise sharply in those patients who do not have any signs of cardiovascular pathology and damage of myocardial cells. And the more the renal function is suppressed (i.e., the lower the filtration rate is), the higher the concentration of cardiac troponins in the bloodstream rises [190–192]. In other pathological conditions that are accompanied by inhibition of the filtration rate, for example, in sepsis, serum levels of cardiac troponins are positively correlated with serum creatinine levels [193, 194], which also accumulate due to a decrease in the filtration capacity of nephrons. From a pathogenetic point of view, any conditions accompanied by a drop in the filtration rate can contribute to the accumulation of troponins. This fact, of course, should be taken into account by medical practitioners when interpreting the results.

Recent clinical studies by several research groups can be considered as valuable evidence of the existence of a mechanism for the elimination of cardiac troponins across the filtration barrier [34, 67]. A key feature of these studies is the use of highly sensitive troponin immunoassays, which can detect small concentrations (from several ng/L to several tens of ng/L) of cardiac troponins in urine. According to these studies, it is also noteworthy that there is a possibility of noninvasive assessment of myocardial damage in arterial hypertension and diabetes mellitus [34, 67], which is very convenient for nonhospital and outpatient settings. This will allow monitoring the patient's condition, assessing the prognosis, and, on its basis, choosing/correcting the tactics of further management of patients, including their treatment. However, it should be noted that these methods have not yet been completely validated and research work in this direction should be continued before introducing new noninvasive methods for diagnosing and monitoring cardiovascular pathologies in routine clinical practice.

One of the key and very labile factors affecting the glomerular filtration rate (including the rate of removal of cardiac troponins from the bloodstream) is blood pressure. So, with a decrease in blood pressure, the filtration rate will slow down and the degree of removal of cardiac troponins from the bloodstream will decrease. This mechanism, in particular, can contribute to the fact that the molecules of cardiac troponins will increase much higher and circulate in the bloodstream for longer in pathological conditions accompanied by a sharp drop in blood pressure. This can be typical for large-focal myocardial infarctions, which are often accompanied by a sharp decrease in blood pressure (cardiogenic shock), and the degree of increase/duration of circulation of cardiac troponins in the bloodstream can be considered as a prognostically unfavorable sign [195]. With an increase in blood pressure, the filtration rate may increase, and more cardiac troponin molecules will be filtered from the bloodstream into the urine. The evidence for a possible role of this mechanism comes from a clinical study showing that urinary troponin levels are higher in hypertensive patients than in those with normal blood pressure or those taking antihypertensive drugs [67].

Another way of cardiac troponins removal is associated with the activity of the reticuloendothelial system, the cells of which capture protein molecules of cardiac markers from the bloodstream and cause their intracellular proteolytic cleavage [187, 188, 196, 197]. The clinical significance of this mechanism for removing cardiac troponins (as opposed to the mechanism for removing cardiac troponins through the glomerular filter) is difficult to judge, since there are no similar well-controlled clinical studies confirming the possibility of a significant increase in serum levels of cardiac troponins in case of the reticuloendothelial system dysfunction. In addition, in contrast to renal failure, dysfunctions of the components of the reticuloendothelial system are much less common.

As noted earlier, the proteolytic cleavage of troponin molecules in the bloodstream is an extremely understudied mechanism for the elimination of cardiac troponins. As a result of this mechanism, a large number of small fragments of cardiac troponins are formed, which can be immunoreactive (can interact with antibodies and be detected by immunoassays) and nonimmunoreactive fragments (which will not interact with antibodies). From the point of view of laboratory diagnostics, nonimmunoreactive fragments of troponins can be considered already removed from the bloodstream, since they will not bind to antibodies and thus will not have any effect on the result of laboratory diagnostics of myocardial infarction or any other pathology. To elucidate the mechanism of cardiac troponin removal by proteases, well-controlled basic research is needed to thoroughly investigate the role of individual serum proteolytic enzymes in the degradation of cardiac troponin molecules in the bloodstream.

Thus, there can be distinguished 3 main mechanisms of elimination of cardiac troponins from the bloodstream: (1) elimination (filtration) of cardiac troponins through the glomerular barrier, (2) removal of cardiac troponins from the bloodstream by cells of the reticuloendothelial system, and (3) proteolytic cleavage of cardiac troponin molecules and/or their fragments in the bloodstream to nonimmunoreactive forms. Taking into account the analysis of the literature, the main mechanism for the removal of cardiac troponins, in my opinion, is the elimination of troponins through a three-layer filtration (glomerular) barrier. This mechanism can have a significant impact on the diagnostics of cardiovascular diseases, including myocardial infarction, since impaired removal of cardiac troponins from the bloodstream is often accompanied by a significant increase in serum levels of cardiac troponins. In addition, many patients have comorbid pathologies, among which kidney damage (chronic renal failure) is relatively common. Many other common diseases, for example, diabetes mellitus, sepsis, are also often complicated by renal failure. Thus, they may increase serum levels of cardiac troponins in patients having no signs of cardiovascular diseases.

Removal of cardiac troponins from the bloodstream by glomerular filtration may have an important impact on rapid algorithms for diagnostics/exclusion of myocardial infarction. Thus, the research group led by Kavsak reported that the currently established upper threshold levels of troponins (99th percentile) for the diagnostics/exclusion of myocardial infarction can be used only for patients with an optimal glomerular filtration rate (≥90 mL/min) [198]. In patients who have lower glomerular filtration rate values, cardiac troponin levels will increase due to impaired elimination, which can lead to overdiagnosis of myocardial infarction if medical practitioners do not take renal function (filtration rate value) into account. Thus, it is necessary to stratify the threshold values of cardiac troponins taking into account different values of the filtration rate and, in particular, to develop special algorithms for diagnostics/exclusion of myocardial infarction for patients who suffer from concomitant chronic renal failure.

Finally, the filtration of troponin fragments through the blood-brain barrier into the cerebrospinal fluid and through the blood-salivary barrier into saliva can be considered as additional potential mechanisms for the removal of cardiac troponins. As evidence of the existence of these mechanisms, one can consider studies [35–37, 68, 74–76], which reported on the detection of cardiac troponins in the cerebrospinal fluid and saliva. The investigation of cardiac troponins in the cerebrospinal fluid can be used in forensic medicine, and the investigation of cardiac troponins in saliva—in clinical practice for diagnostics and monitoring of cardiovascular pathologies, including myocardial infarction. Overall, more research is needed to validate these diagnostic capabilities.

### 2.6. Circadian Rhythms of Cardiac Troponins: Possible Mechanisms of Formation and Diagnostic Role

The activity of many systems (organs, tissues, and cells) of our body changes cyclically during the day (with the change of day and night), which is commonly called circadian or diurnal rhythms. Circadian rhythms are an evolutionarily developed mechanism necessary to maintain optimal functioning of the body and adapt to changing environmental conditions [199].

Due to the fact that the tissues and cells of our body change, there is a change in the concentration of a number of molecules (for example, hormones, metabolic products), which are produced or metabolized by these tissues and cells. Many of these molecules are laboratory biomarkers, the concentration of which is used to diagnose diseases [200, 201]. This must be taken into account in routine clinical practice, since changes in the concentration of biomarkers caused by natural circadian rhythms can be mistakenly interpreted as diagnostic signs and, accordingly, lead to diagnostic errors. Certain hormones, the release of which varies from day to night, can affect a number of other laboratory parameters that must also be considered when interpreting laboratory diagnostic results.

Recent clinical studies have reported that bloodstream levels of cardiac troponins are dependent on circadian rhythms. These studies used highly sensitive troponin immunoassays able to detect small fluctuations in the concentration of cardiac troponins in the bloodstream (at the level of several ng/L) [46, 47, 202, 203]. For example, Klinkenberg et al. revealed changes in troponin T concentration (detected by a highly sensitive method) in patients without signs of cardiovascular diseases. At the same time, the maximum levels of troponins were recorded in the morning (16.2 ng/L at 8 : 30), and the minimum—in the evening (12.1 ng/L at 19 : 30). In addition, when analyzing the hourly curve of serum levels of cardiac troponins, the researchers found very regular and gradual changes: for example, from the maximum morning concentrations of troponins there was a gradual decrease to the evening (minimum) concentrations of cardiac troponins, and then there was a gradual increase in concentrations to the maximum morning values [202]. However, the researchers noted that such relatively minor circadian fluctuations in troponins would not have a significant impact on diagnostic algorithms for myocardial infarction, but should be considered for screening purposes. The levels of cardiac troponin I (also detected by a highly sensitive immunoassay) changed over a 24-hour period by no more than 1 ng/L, i.e., had no significant circadian rhythms [202]. However, this study investigated the circadian rhythms of troponins only in healthy people, but in conditions of concomitant pathologies (especially with damage to those organs that affect the metabolism of cardiac troponins), fluctuations in the circadian rhythms of troponins can be much more pronounced. Thus, in patients with concomitant chronic renal failure, troponin T and troponin I concentrations changed more significantly during the day. van der Linden et al. [203] reported that the maximum fluctuations in troponin T concentration in a patient with chronic renal failure during the 24-hour investigation period were about 50 ng/L, while the fluctuations in troponin T levels during one hour were about 20 ng/L, which, by the way, is a very significant contribution to the laboratory diagnosis of myocardial infarction. So, for example, if we take into account modern algorithms for diagnostics of non-ST-segment elevation myocardial infarction (Table 1) [29] (where the change in the levels of cardiac troponins within 1-2 hours by only 5–10 ng/L is diagnostically significant), we can say that troponin T circadian rhythms may affect the diagnostics of myocardial infarction and contribute to overdiagnosis [203]. Troponin I levels showed slightly higher fluctuations in concentration during the day compared to the study by Klinkenberg et al. [202], however, they would not reach the thresholds of 5–10 ng/L and thus would not have a significant effect on one- and two-hour algorithms of myocardial infarction diagnostics.

The precise mechanisms of the formation of circadian rhythms of cardiac troponins are unknown, however, it can be assumed that they will be associated with changes in the functional activity of those organs, tissues and cells that can somehow affect the metabolic pathway of cardiac troponins, in particular the stages of their release into the bloodstream, the stage of circulation (for example, the effect on the activity of proteolytic enzymes that cause the cleavage of troponins in the bloodstream) or the elimination stage (for example, the effect on the functional state of the kidneys). Among the most probable mechanisms for the formation of circadian rhythms of cardiac troponins, in my opinion, there are circadian fluctuations in the activity of the cortex and medulla of the adrenal glands, of the thyroid gland, and the activity of enzymes of the hemostatic system [54, 204–208]. A possible rationale for the formation of circadian rhythms is that peak troponin concentrations occur in the morning period, being the period of the maximum activity of the adrenal glands (producing elevated levels of catecholamines, cortisol), the thyroid gland (producing thyroid hormones, which can enhance the effects of catecholamines on myocardial cells). The increased activity of these organs also coincides with their main effects on the cardiovascular system, namely, in the morning period, patients have the highest heart rate, and the blood pressure is higher than in the evening-night period. In general, the increased activity of these organs is a kind of adaptive and evolutionary developed mechanism, which is necessary to maintain the period of wakefulness. However, we should take into account the negative impact of these organs and their metabolic products (for example, catecholamines and cortisol) on myocardial cells. The evidence of the adverse effect of cortisol on myocardial cells is a clinical study that demonstrates that increased levels of the stress hormone (cortisol) are associated with increased levels of cardiac troponin T [165]. In addition, a number of researchers associate the increased high activity of the sympathoadrenal system with a larger size of the focus of myocardial necrosis in myocardial infarction, the incidence of acute cardiovascular diseases and an unfavorable prognosis [209–217].

A possible explanation of the reason for the fact that the circadian rhythms of troponin T are more significant than the circadian rhythms of troponin I consists in their biochemical features, in particular, the volume of the cytoplasmic fraction of troponin T is almost twice the volume of the cytoplasmic fraction of troponin I (approximately 7–8% versus 3–4%) [53, 54]. Thus, the cytoplasmic fraction of troponin T is more “mobile” and can be released into the bloodstream with an increase in the effect of a number of factors on the myocardium. There is a need for further clinical studies validating the circadian rhythms of cardiac troponins and their effect on the diagnostics of cardiovascular diseases, including myocardial infarction, and for fundamental research clarifying the molecular mechanisms of the formation of circadian rhythms of cardiac troponins.

## 3. Conclusion

The metabolic pathway of cardiac troponins includes three main stages (release of troponins from myocardial cells, circulation of cardiac troponins in blood plasma, and removal of cardiac troponins from the bloodstream), each of which can have a very significant effect on serum levels of cardiac troponins, i.e., on their diagnostic value.

It should be noted that many new views on the metabolism and diagnostic value of cardiac troponins (in particular, the role of circadian rhythms, gender- and age-related characteristics of concentrations, and the possibility of detecting troponins in urine and saliva) were formed as a result of an increase in the sensitivity of troponin immunoassays.

Unfortunately, today many stages of the metabolic pathway of cardiac troponins and factors influencing the metabolic pathway of cardiac troponins are extremely poorly understood and are hypothetical and/or contradictory. In particular, the specific mechanisms of the release of cardiac troponins from the myocardium into the bloodstream as affected by physiological conditions and characteristics (physical exertion, stress, and circadian fluctuations in the activity of organs and tissues that influence the release of cardiac troponin molecules) and nonischemic pathologies, which are often accompanied by an increase in the concentration of cardiac troponins in the bloodstream, are little known. And factors affecting the circulation of cardiac troponin molecules in the bloodstream, in particular enzymes involved in the metabolism (fragmentation) of troponin molecules, remain unknown. The mechanisms of filtration (transport) of cardiac troponin molecules from the bloodstream to other biological fluids are not investigated, and, accordingly, these possibilities of noninvasive diagnostics have not been validated. Thus, the study of the metabolic pathway of cardiac troponins and potential factors influencing it is a relatively large and poorly studied area for further research that is needed to optimize diagnostics and validate new diagnostic capabilities.

## Figures and Tables

**Figure 1:** Interpretation of possible reasons for myocardial injury and increase in cardiac troponin serum levels.

**Figure 2:** Metabolic pathway of cardiac troponins.

**Table 1:** Current diagnostic algorithms for confirmation/exclusion of NSTEMI (0 → 1 hour and 0 → 2 hours), approved by the ESC [29].

One-hour NSTEMI diagnostic algorithm					
Troponin immunoassay, company (manufacturer)	Biomarker concentration that indicates an extremely low probability of an NSTEMI diagnosis (ng/L)	Biomarker concentration that indicates a low probability of an NSTEMI diagnosis (ng/L)	Changes in biomarker concentration after 1 hour at which a diagnosis of NSTEMI should be excluded (ng/L)	Biomarker concentration that indicates a high probability of an NSTEMI diagnosis (ng/L)	Changes in biomarker concentration after 1 hour at which a diagnosis of NSTEMI should be confirmed (ng/L)
Cardiac troponin T (Elecsys; Roche)	<5	<12	<3	≥52	≥5
Cardiac troponin I (Architect; Abbott)	<4	<5	<2	≥64	≥6
Cardiac troponin I (Centaur; Siemens)	<3	<6	<3	≥120	≥12
Cardiac troponin I (Access; Beckman Coulter)	<4	<5	<4	≥50	≥15
Cardiac troponin I (Clarity; Singulex)	<1	<2	<1	≥30	≥6
Cardiac troponin I (Vitros; Clinical Diagnostics)	<1	<2	<1	≥40	≥4
Cardiac troponin I (Pathfast; LSI Medience)	<3	<4	<3	≥90	≥20
Two-hour NSTEMI diagnostic algorithm					
Troponin immunoassay, company (manufacturer)	Biomarker concentration that indicates an extremely low probability of an NSTEMI diagnosis (ng/L)	Biomarker concentration that indicates a low probability of an NSTEMI diagnosis (ng/L)	Changes in biomarker concentration after 2 hours at which a diagnosis of NSTEMI should be excluded (ng/L)	Biomarker concentration that indicates a high probability of an NSTEMI diagnosis (ng/L)	Changes in biomarker concentration after 2 hours at which a diagnosis of NSTEMI should be confirmed (ng/L)
Cardiac troponin T (Elecsys; Roche)	<5	<14	<4	≥52	≥10
Cardiac troponin I (Architect; Abbott)	<4	<6	<2	≥64	≥15
Cardiac troponin I (Centaur; Siemens)	<3	<8	<7	≥120	≥20
Cardiac troponin I (Access; Beckman Coulter)	<4	<5	<5	≥50	≥20
Cardiac troponin I (Clarity; Singulex)	<1	To be determined	To be determined	≥30	To be determined
Cardiac troponin I (Vitros; Clinical Diagnostics)	<1	To be determined	To be determined	≥40	To be determined
Cardiac troponin I (Pathfast; LSI Medience)	<3	To be determined	To be determined	≥90	To be determined

**Table 2:** Biological fluids in which the molecules of cardiac troponins are detected and the diagnostic value.

Biological fluid	Diagnostic value of cardiac troponins	Sources
Blood (whole, serum, plasma)	It is the main biological fluid used to diagnose myocardial infarction and assess the prognosis of patients suffering from nonischemic cardiac (myocarditis, Takotsubo syndrome, cardiomyopathies, etc.) and noncardiac (sepsis, renal failure, neurogenic pathologies, etc.) pathologies that cause damage to myocardial cells	[24–28]
Urine	Molecules of cardiac troponins can be detected in this biological fluid via highly sensitive test systems. Increased troponin levels have a high prognostic value in diabetes mellitus and arterial hypertension. The method of obtaining this biological fluid is noninvasive, which has a number of advantages over the use of blood. It should be noted that the possibilities of examination of highly sensitive troponins in urine are still poorly studied and have not been finally validated. Further research is needed before the introduction of this method into clinical practice	[34, 67, 69]
Oral fluid	The levels of cardiac troponins in oral fluid increase in myocardial infarction and moderately correlate with serum troponin levels; therefore, further study of this area of noninvasive diagnostics is very promising	[35–37, 68]
Pericardial fluid and cerebrospinal fluid	Molecules of cardiac troponins are detected in pericardial fluid and cerebrospinal fluid via moderately sensitive and highly sensitive test systems and, according to some studies, may correlate with serum levels of cardiac troponins. Increased troponin levels in these biological fluids may reflect the degree of myocardial damage and may be used in forensic medicine to determine the cause of death. However, due to the relative paucity of such studies, further investigation of these possibilities is necessary	[72–76]
Amniotic fluid	Cardiac troponin molecules can be detected in amniotic fluid via moderately sensitive and highly sensitive immunoassays. Increased troponin levels may indicate chronic fetal hypoxia, abnormal development of the cardiovascular system and fetal myocardial injury, and an increased risk of fetal death during the intrauterine growth period. However, it is worth noting that such studies are few in number. Further research is needed to clarify the diagnostic capabilities of amniotic fluid	[77–80]

**Table 3:** Release of cardiac troponins from myocardial cells: mechanisms and diagnostic value.

Mechanism	Diagnostic value
Myocardial cell necrosis	This is the main proven mechanism underlying the increase in cardiac troponins in myocardial infarction. Cardiomyocyte necrosis will result in the release of all molecules (biomarkers) from the cell into the bloodstream
Release of cardiac troponins as a result of the processes of regeneration and renewal of myocardial cells	The renewal of myocardial cells gradually occurring throughout life, hypothetically, may be associated with normal (less than the upper limit of the 99th percentile) concentrations of cardiac troponins in the bloodstream
Release of cardiac troponins as a result of apoptosis of myocardial cells	It has been proven that apoptosis of cardiomyocytes (without signs of necrosis) is accompanied by an increase in the serum concentration of cardiac troponins. Thus, any physiological (physical activity, old age) and pathological (heart failure, arterial hypertension, chronic obstructive pulmonary disease, etc.) conditions that enhance apoptosis may be accompanied by the release of cardiac troponins from cardiomyocytes and an increase in serum levels
Release of cardiac troponins as a result of the formation of membrane vesicles on the surface of myocardial cells	Membrane vesicles (blebbing vesicles) formed on the surface of the plasma membrane of cardiomyocytes, hypothetically, may contain cytoplasmic proteins, including cardiac troponins. The number of membrane vesicles increases during ischemia of myocardial cells and may be associated with the release of cardiac troponins into the bloodstream
Intracellular proteolytic degradation of cardiac troponin molecules into small fragments and the release of the latter through the intact membrane of myocardial cells	Molecules of cardiac troponins can be fragmented/destroyed by the action of certain proteolytic enzymes: calpain, thrombin, and matrix metalloproteinases. As a result of the action of these enzymes, there can form small fragments of troponin molecules, which, due to their size, have a higher probability of release from the cell. This mechanism may have high clinical significance: for example, all those physiological and pathological conditions and/or drugs that affect the activity of these proteolytic enzymes can also affect the release of cardiac troponins and their concentration in the bloodstream
Release of cardiac troponins as a result of increased membrane permeability of myocardial cells	An increase in the release of cardiac troponin molecules into the bloodstream is observed in case of an increase in the membrane permeability of myocardial cells, which is characteristic of myocardial ischemia, an increase in preload and stretching of the heart wall
Release of cardiac troponins as a result of small-scale (subclinical) necrosis of cardiomyocytes	The death of a small number of cardiomyocytes may not manifest itself clinically and instrumentally (since these are relatively low-sensitivity methods), but highly sensitive methods of detection can register such subclinical lesions. Possible causes of subclinical necrosis of cardiomyocytes are ischemia, inflammatory-toxic processes, and imbalances in the neuroendocrine system
Release of cardiac troponins from noncardiac cells	This is a controversial mechanism of increased levels of cardiac troponins in the bloodstream. In the literature, there are works confirming the expression of cardiac troponins in skeletal muscle tissue in patients with chronic renal failure and hereditary skeletal myopathies, as well as studies that refute this hypothesis
